The article "Slime-Groove Drag Reduction Characteristics and Mechanism of Marine Biomimetic Surface" was published in 2022. Journal: Appl Bionics Biomech.

# Slime-Groove Drag Reduction Characteristics and Mechanism of Marine Biomimetic Surface

**DOI:** 10.1155/2022/4485365

**Published:** 2022-03-14

**Authors:** Muhan Yan, Yunqing Gu, Longbiao Ma, Jianxing Tang, Chengdong He, Junjun Zhang, Jiegang Mou

**Affiliations:** ^1^College of Metrology & Measurement Engineering, China Jiliang University, Hangzhou 310018, China; ^2^Zhejiang Engineering Research Center of Fluid Equipment & Measurement and Control Technology, Hangzhou 310018, China; ^3^Nanfang Smart Water Technology Co., Ltd, Hangzhou 311106, China

## Abstract

With the development of science and technology, energy consumption and demand continue to increase, and energy conservation and consumption reduction have become the primary issue facing the world. Improving the energy efficiency of ships not only helps reduce fuel consumption but also reduces carbon dioxide emissions, which is an important guarantee for the green development of the ocean and the maintenance of ecological balance. Through natural selection and adaptation to the environment after evolution, the body surface of organisms generates a variety of ways to resist adhesion and resistance of Marine organisms. Through the study of fish organisms, it is found that the body surface of general fish has mucus, which can effectively reduce the friction resistance of the body surface of fish subjected to seawater. In addition, the grooves on the body surface also help to reduce the resistance between swimming organisms and fluids. Based on the principle of bionics, the drag reduction characteristics and mechanism of fish surface mucus were analyzed. The drag reduction mechanism of bionic nonsmooth surface is analyzed from the aspect of body surface structure. On the basis of the two approaches, the characteristics and mechanism of slime and groove codrag reduction on the surface of Marine organisms were discussed in depth, so as to obtain a better new drag reduction method and provide reference for subsequent related research.

## 1. Introduction

Energy crisis has become a thorny problem all over the world. Global energy demand and consumption is increasing day by day, the concept of low-carbon environmental protection has been deeply rooted in the people, and energy saving and consumption reduction have always been one of the important issues concerned by researchers. Since entering the 21st century, Marine strategy has become the core national interest [1], and marine economy and maritime national defense have become the most important development strategies of some major powers. Ship is an important strategic transportation material in the ocean [2], as global freight volumes increase [3]; ship-derived greenhouse gas emissions are expected to increase to 250 percent by 2050 from 2012 levels. Unchecked, it is expected to account for 17% of global CO_2_ emissions by 2050, up from around 2% at present [4]. Because ships working in the water for a long time need to carry enough fuel, but in the general ship sailing process, there will be some resistance, of which the boundary layer resistance accounts for about 70% to 80% of the total resistance [5]; in high-speed ships, the boundary layer resistance accounts for 40% of the total resistance [6]; in addition, the underwater instrument must overcome the drag caused by fluid pressure and friction between the fluid and the wall. If the surface water resistance is reduced by about 10%, the ship's speed and navigation will increase by about 3.57% [7]; therefore, the fuel carried cannot fully meet the navigation, resulting in excessive energy consumption. Hard-shelled fouling is an important factor leading to a large increase in the friction resistance of ships [8], which leads to an increase in the fuel consumption of ships. Therefore, the best way to reduce the friction resistance is to treat the hull and apply some preventive measures, such as antiadhesion coating, to minimize the physical and biological roughness.

There are two ways to reduce resistance: one is to achieve it through common fluid drag reduction methods, mainly including structural optimization, bionic nonsmooth surface, surface coating, microbubbles, vibration drag reduction, and jet drag reduction [9–16]. Another idea is to reduce drag by reducing attachments. Traditional drag reduction methods are difficult to achieve in the vast ocean, and for the protection of the Marine environment, the traditional antiadhesion coating is also easy to pollute the Marine environment. Therefore, the learning and understanding of biological characteristics of long-term evolution in nature through the principles of bionics provide a lot of enlightenment for human beings to solve engineering problems [17]. As early as in ancient times, organisms have been optimized through long time evolution and natural selection, which not only better adapt to nature but also adapt to external systems in the best form. Bionics attempts to mimic the functions of organisms in nature in terms of technology, analyze biological processes and structures, and apply their analysis to future designs. This idea builds a bridge between biology and engineering technology and provides help to solve engineering problems. The task of bionics is to study the excellent ability of a biological system and its generation principle and transplant these principles into engineering technology, invent superior performance instruments and new technical equipment, design and manufacture devices and machines and mechanical instruments, and create new technology, so as to serve human production and life. Simulation of the special characteristics of biology has become one of the important ways to develop high and new technology in modern times, providing new design ideas and broadening ideas for engineering technology research. In bionics, bionic drag reduction involves taking techniques from delicate structures that reduce drag in nature and then simulating them for use in instruments. From the perspective of the most intuitive animal surface, it is generally believed that the smoother the surface of an object, the less friction it will generate and the less friction it will suffer. However, researches on the skin of tuna [18], shark [19], dolphin [20], and other animals have found that they all have a microgroove structure on their surfaces. They can be made to greatly reduce friction under certain turbulent conditions. An in-depth study of the above animals shows that the microgroove structure similar to the surface of shark scales can freely rotate in the range of 50°; Figure 1 shows the histological section [21–23], so as to adapt to the direction of turbulent flow in different directions, which can reduce the resistance. Similarly, inspiration can also be obtained from plants. For example, the superhydrophobic surface of lotus leaves [24] enables them to have extremely water repellency, that is, there is very little resistance between water and the skin of lotus leaves, as shown in Figure 2.

The bionic drag reduction method not only has the bionic nonsmooth surface drag reduction and groove drag reduction, and the method of biomimetic polymer additives [25] is also a very typical bionic drag reduction method; groove drag reduction is modelled on the geometry of a certain scale of the groove of turbulent drag reduction, a bionic polymer additive method using some kind of mucus materials coated to the surface to drag reduction. After years of research, it is found that bionic drag reduction has the advantages of good drag reduction effect and strong designability, which has been a hot spot in the field of drag reduction in recent years. Derived from the advantages of biological drag reduction, this paper firstly studied the slime mechanism of Marine fish from the drag reduction characteristics of slime, combined with the analysis of the “water-catching” effect of the groove and its mechanism, and finally analyzed the synergistic drag reduction mechanism of slime and groove, so as to reveal the drag reduction mechanism of slime and groove characteristics on the surface of fish organisms.

## 2. Bionic Mucus Drag Reduction Analysis

Marine biological adhesion on ship resistance affects the ship speed and can increase the body weight, leading to increase fuel consumption, although existing prevention coating can increase the efficiency of navigation of ships, but at the same time has a certain negative impact on the Marine environment, such as some antifouling (AF) coating will have a great impact on Marine mammals [26], increase tin content in the ocean, and damage the Marine ecosystem. According to the study, it can be found by observing Marine fish that the surface of fish can produce mucus, which makes it difficult for Marine organisms to adhere to its body surface. Studies have found that the mucus secreted by fish is a highly multifunctional material [27], which plays different roles in many aspects, such as respiration, ion and osmotic regulation, and reproduction. In terms of fluid dynamics, in addition to protecting the body, fish mucus is also commendable in reducing resistance [28]. Dean and Bhushan [29] prepared biomimetic mucus, studied its drag reduction characteristics, and found that mucus containing natural mucus and polyethylene oxide would produce a drag reduction phenomenon similar to fish mucus.

### 2.1. Mucus Drag Reduction Mechanism

Fishes in the ocean have an inherent slime layer, which can not only prevent parasites and bacteria but also reduce the surface resistance of fish when they swim [30, 31]. Loaches are a kind of freshwater fish, and their body surface is covered with a mucous layer. When the loaches (rice field eel) and other organisms in the mud are pressed or scratched, the mucous layer on their surface will be obtained, especially the mucous is easy to attach to the pressuring object, indicating that the mucous has good self-viscosity. In addition, loaches have a mucus layer with weak gel structure formed by mucin glycoprotein, which is secreted by mucinous adenosine cells of the scale [32]. Since the soft tissue of the loach epidermis is rarely seen, the loach epidermis can be observed through dermo scope. Dark-field optical coherence tomography (OCT) imaging was used to conduct real-time imaging of the cross-sectional microstructure of the transverse region of flat, concave, and convex loach skin, as shown in Figure 3(a). After studying the morphology of epidermal surface tissue, it can be seen that mucous secretion is attributed to the interaction between the lower scale and mucous gland cells during the bending movement of scales. As shown in Figure 3(b), mucous gland cells secrete mucous at a high speed. When loaches bend, the sharp edge of the scale surface also stimulates the mucous gland cells. When the mucous layer reaches a certain thickness, the cells stop secreting mucous. Loaches can secrete mucus even when they are not bending, because mucosae cells secrete mucus when stimulated by externally induced stress, such as environmental pollutants.

Studies on the mucous of loaches found that the main component of mucous is water, and water accounts for more than 99% of the total weight, while other components including mucins, proteins, sugars, lipids, and inorganic salts only account for about 0.5% [33, 34]. According to studies on most fish, transient network structures can be found in all types of mucus, as shown in Figure 4, which is the root of mucus drag reduction [35]. The pH of the skin mucus of loach is neutral, and the solid content is between 0.5 wt% and 1 wt%. Therefore, the mucus can be regarded as a viscoelastic fluid. When the external fluid velocity increased, the storage and loss of loach mucus increased, but the storage was greater than the loss. When the external strain increases greatly, the physical state of the mucus appears to be very similar to that of a liquid rather than a gel, but strain disappears, and the mucus immediately reverts to its gel structure. This suggests that there is a reversible interaction between the structure of the mucus to maintain the state. According to rheological studies, loach skin mucus is a weak gel, so it is that the mucus is a flowing liquid under nonoscillation scanning and shows solid rheological behavior under oscillation scanning [33]. If you take only the nonaqueous substances in the mucus and put them in water, the nonaqueous substances will absorb more than 100 times their own weight in water, restoring the mucus to its weak gel state. Therefore, it can be inferred that there is a highly hydrophilic gel-forming substance in the skin mucus of loach, which is a mucilaginous glycoprotein. According to studies, when the mucus is adsorbed on the hydrophobic surface, it has antifouling and lubrication functions [34].

Mucin is mainly formed by bonded biopolymers [36]. Amphiphilic polymer nanocomposites are the main pollution-resistant polymer coatings. These materials have low polymer-water interface energy. When a biological starter is attached to the surface, the high degree of hydration increases the energy loss of water removal; therefore, the surface is resistant to protein adsorption and sedimentation of contaminated organisms [37]. Several hydrophilic polymer nanocomposite coatings are as follows: polyethylene glycol (PEG), hydrogels, amphoteric ions, and hyperbranched polymers. Pegylated materials are used because of their strong AF tendency to bind cells and proteins. Polyethylene glycol is nontoxic, highly hydrophilic, and neutral charged. PEG has a weak alkaline ether connection and a reduced interface energy with water (5 mJ/m^2^), which contributes to its good AF performance [38]. Maximizing surface hydrophilicity and reducing attraction (caused by hydrogen bonding with water) with contaminated communities are key to PEG. AF efficiency of long-chain polyethylene glycol is higher than that of oligomer (ethylene glycol) (OEG). PEG prevents spore and larva attachment, and the OEG-modified surface reduces spore and larva adhesion so that PEG is easily released with a small hydrodynamic force, as shown in Figure 5.

In addition, studies of fish slime in the ocean have revealed that there are two main ideas trying to explain the mechanism of slime resistance reduction in fishes: (1) the mucus of polymer slightly soluble in water weakened the turbulent boundary layer under the condition of vibration, so that the fish in a relatively short period of time consumption is low, greatly reducing the resistance when the fish swim; this is similar to the use of the additive drag reduction method [40]; this type of drag reduction method to polymer or surfactant in water injection pipe, in order to realize the resistance, is reduced; this drag reduction method can achieve a maximum drag reduction rate of about 80% with strong drag reduction effect and low investment cost [41], and the polymer used is nontoxic and harmless. (2) It was found that the long-chain polymers in the mucus reduced the pressure gradient and correspondingly reduced the friction. This phenomenon shows that the fish's skin mucus exhibits gelatinous characteristics. Fish skin mucus is mainly secreted by epidermal goblet cells, and its main components are water plus proteins, sugars, polysaccharides, and lipids as secondary components [42], which can interact to form gel structures. Similarly, shark mucus secreted by shark skin surface also plays a positive role in reducing resistance. Shark mucus is mainly composed of water-soluble polymers and insoluble lipids. Shark mucus secreted by shark will quickly swell and become sticky and eventually form mucus, and the maximum reduction rate of mucus resistance can reach 80% [43]. Mucus separates sharks from the water environment and forms a boundary layer. Particularly in areas with strong turbulence, local dissolution of mucus can attenuate the vibration of a turbulent boundary layer and reduce the resistance of swimming to the maximum extent [44].

### 2.2. Mucus Properties

The surface of some Marine organisms is not easy to be attached by defiled organisms and can effectively reduce their swimming resistance in water, showing good antifouling and drag reduction ability. The reason is that its mechanism includes chemical antifouling mechanism and the synergistic effect of various antifouling mechanisms, which provides bionic objects for the development of bionic drag reduction materials and antiresistance mucus, as well as an important basis for the development of bionic antifouling materials [45]. At present, antifouling (AF) coating strategies are mainly used in bionic mucus antiadhesion coatings. Marine AF coating strategies can be divided into two categories: one is chemical coating and the other is pollution releasing coating. To make the coating more strongly adhere to the hull, polymers such as crosslinkers are needed.

#### 2.2.1. Chemical AF Coating

Chemical antifouling coating technology is mainly based on the release of fungicides to inhibit the adhesion of Marine organisms [46]. Chemical antifouling coating of drag reduction technology can be traced back to the original [47] in 1625, but until the 1860s, but the actual use of paint is the main material of arsenic, copper, and mercury compounds as the agent, resin as the basic material of thermoplastic and cold plastic paint; since the 20th century, antifouling paint research is developing rapidly; but until 1970, copper and copper compounds (mainly cuprous oxide) have still been the main antifouling agent of antifouling paint, and sometimes with mercury oxide and organic metal compounds such as lead, mercury, arsenic, zinc, tin, and other antifouling agents. In the middle of the 1960s, the invention of tributyltin (TBT) self-polishing antifouling coating marked a new height of antifouling technology, and its wide application brought huge economic benefits to shipping industry. At first, TBT was incorporated into the traditional antiadhesion coating, mainly using surface poisons transmitted by a soluble matrix to inhibit the growth of Marine organisms, as shown in Figures 6(a) and 6(b). However, due to the difficulty in controlling the toxicity and number of poisons released through a soluble matrix, it is gradually replaced by self-polishing copolymer (SPC) coatings, in which TBT copolymer provides a biocide, but this provides a paint substrate, which is hydrolyzed in seawater and releases TBT. As the hydrolysis process increases, an unstable surface layer is exposed. Finally, a new layer of active coating appears, as shown in Figure 6(c). Although these measures do not prevent the settlement of fouling organisms, they can reduce the adhesion strength and also cause Marine organisms to shed with resistance when the hull is running, as shown in Figure 6(d).

However, AF coating can seriously affect nonobjective organisms, such as dolphins [49]. Organotin antifouling agents have good antifouling effects, but only 1/10^10^ organotin in seawater is enough to distort some Marine organisms and inhibit the reproduction of Marine organisms, and the Marine organisms containing organotin are not suitable for consumption. When using an antifouling agent containing cuprous oxide, when the concentration of cuprous oxide in seawater is 0.68 mg/L, it can inhibit the growth of various algae. When the concentration is 25~50 mg/L, it can poison diatoms and then bring harm to fish that feed on diatoms. In addition, AF coating technology may lead to accelerated corrosion of metal surface or damage of the protective layer on the hull, and it will seriously affect the water quality of the ocean, resulting in a double increase in the cost of sewage treatment.

#### 2.2.2. Contamination Release Coating

Fouling release coatings (FRCs) inhibit biological pollution or enhance pollution release (FR) without involving chemical reactions [50]. The dirt release coating is a fungicide-free coating that achieves AF performance in a dual mode of nonsticky behavior and dirt release performance. Self-cleaning of FRCs during ship sailing is shown in Figure 7. By driving the boat to a certain speed, the biological coating cleans itself at different speeds. In addition, the smoothness and hydrophobicity of the FRC can reduce the ship's drag during navigation, thus reducing fuel consumption and carbon dioxide emissions. However, such coatings also have the disadvantage of being difficult to apply directly to antiseptic substrates. Therefore, a binding coating is required to promote adhesion between the FRC and the corrosion-resistant substrate [51]. And only when applied to ships with high frequency of movement and fast movement (>15 knots) can the FR technology show better performance. Therefore, the application of FRCs is relatively limited, which is not suitable for low-speed cruising and long time berthing in ports. Therefore, it is necessary to find an environmentally friendly coating [52] that has no impact on the ecological environment.

For FRCs, binding coatings are required to stick to the hull, but due to the contamination, bionics is needed to find a strong adhesive that is both efficient and Marine friendly. The preparation of long-chain gels similar to mucin can improve the mechanical properties of gelatin-based hydrogels by EDC/NHS chemical crosslinking [53]. Glutaraldehyde [45], GDTA, and carbodiimide can be used, etc. GTA is one of the most widely used crosslinking agents at present. The synthesis scheme is shown in Figure 8. GTA reacts quickly with the amine groups in gelatin and is relatively inexpensive [54]. And it is found that glutaraldehyde crosslinked gelatin hydrogel can be used to simulate fish mucus, not only as a binding coating but also as a resistance reduction coating on metal matrix.

Biomimetic mucus can also do the job of FRCs. Mucus can be obtained by emulsion polymerization [55]. Polystyrene microspheres with polyethylene glycol branched chains on the surface are mainly prepared by emulsion polymerization. The suspension of microspheres is blended with acrylic polymer emulsion to obtain bionic biological mucus, as shown in Figures 9 and 10. In addition, mucins have large molecular weight, polydispersity, and high degree of glycosylation. The nonglycosylated region is a dimer formed by dimers linked by disulfide bonds, which form a higher dimer. This results in the high molecular weight and polydispersity of secretory mucins, as shown in Figure 11. Highly flexible polyurea is also a very good slime-like drag reduction material, which can be generated by diisocyanate, medium long-chain amino ether, and aromatic steric diamine chain extender.

#### 2.2.3. Enhance the Adhesion of the Coating

For the above two AF coating types, the performance will be reduced due to slow shedding after a long time of use. Therefore, effective adhesion to the hull is an important link. Xue et al. [56] developed a novel polymer crosslinking agent based on photocurable poly(vinyl alcohol) (UV-PVA). The synthesis diagram of UV-PVA is shown in Figure 12. This agent reacts with dopamine methylacrylamide (DMA) to improve its adhesion strength. The adhesive strength of the gel reached 1.87 MPa. Ai et al. [57] photopolymerized trimer by dopamine acrylamide [51], N-isopropylenolamide (NIPAAm), and poly(ethylene glycol)-triacrylate (PEG-TA), as shown in Figure 13. After 2 h and 6 h, the interface adhesion strength was 2.08 ± 0.22 MPa and 2.27 ± 0.33 MPa, respectively. Fan et al. [58] designed a mussel-inspired double-crosslinked tissue adhesive (DCTA) that is easy to use, consisting of dopamine-bound gelatin macrosubstance Fe^3+^ and gene protein. Using cartilage as substrate, the ability of DCTA was measured. The adhesion strength was 194.4 ± 20.7 kPa. White and Wilker [59] designed a biomimetic copolymer family containing DOPA chemical and cationic charges to explore the role of charge in adhesion. The adhesion strength of copolymer is quite high; the combination of catechin-containing phenol monomer (10%) and cationic monomer (7%) reaches 2.8 ± 0.6 MPa. These results show that the adhesive strength of the polymer can be significantly improved by modifying the polymer with catechol groups. Therefore, the hydrogels of DOPA-modified gelatin may combine resistance reduction and strong adhesion ability. The gelatin-DOPA was crosslinked with Fe^3+^ and GTA to synthesize gelatin-3,4-dihydroxyhydrocinnamic acid (gelatin-DOPA). Some similar binding polymer solutions, such as hydrophobic ethoxylated polyurethane and chitosan-polyacrylamide graft copolymer, showed similar effects to loach skin mucus [36]. Similarly, polymers such as polyvinyl pyrrolidone, polyvinyl alcohol, and polyacrylamide can be used to simulate shark slime. Shirahama et al. [60] first studied the composite of surfactant and polymer interaction by electrophoresis. Surfactant molecules adsorbed on the molecular chain of polymer in the form of micellar aggregates, resulting in a synergistic effect, which not only made the adhesion strength higher but also had a better drag reduction effect.

The way long chains of different compounds bind, Zhao et al. [53] used the rotation method to measure the resistance reduction performance of hydrogel coating, coating 1 (gelatin-DOPA-Fe^3+^), coating 2 (gelatin-DOPA-Fe^3+^-GTA-1), coating 3 (gelatin-DOPA-Fe^3+^-GTA-2.5), and coating 4 (gelatin-DOPA-Fe^3+^-GTA-5). The torque values of the control group and the coating group at different speeds were studied, and the contents in Table 1 were obtained.

In addition, the application of nanomaterials [61] to polymers can make nanomaterials have volume effect and surface effect that ordinary polymers do not have and improve the mechanical properties, corrosion resistance, thermal stability, and wear resistance of the matrix. The method of reducing turbulent frictional resistance through polymer additives has been widely used in the direct application of ship drag reduction [62].

## 3. Bionic Groove Surface Drag Reduction Analysis

The bionic drag reduction method is to achieve the drag reduction function by imitating the special ability of organisms and utilizing the structure and functional principle of organisms [63, 64]. For example, the strong drag reduction performance of dolphins reduces the velocity gradient of boundary layer and wall shear stress through adaptive surface, achieving a good drag reduction effect [65]. Nonsmooth surface structure is a typical bionic drag reduction method, which has obvious drag reduction effect, green environmental protection, and good sustainable energy. Nonsmooth surfaces can change the way fluid interacts with the wall. For example, biosimilar pits and other structures can be added to the surface to reduce drag. The high speed of sharks also depends on the special structure of their body surface, and the unique structure of the mantis shrimp's abdomen can reduce resistance and vibration when attacking prey [66].

### 3.1. Bionic Groove Drag Reduction Mechanism

Mantis shrimp is known as the ferocious predator of the sea in the ocean, especially its body is a very perfect hunting machine [67–69]. The structure of mantis shrimp is shown in Figure 14(a). The body is mainly composed of thorax, abdomen, abdomen and appendage [70]. The abdomen is an undulation shape of convex nonsmooth surface [71]. The sixth ventral segment was connected with the caudal segment, which was extracted as the bionic surface, as shown in Figure 14(b). As fluid flows over its body, this structure alters the pattern of water flowing over the shrimp's surface, allowing the shrimp to swim with less resistance. At the same time, obvious vortexes are formed in the low-speed area behind the airfoil. The vortexes are clockwise, the upper direction is the same as the flow direction, and the lower direction is opposite to the flow direction, resulting in the buffering effect of vortexes [72–75]. When fluid flows through the airfoil profile at high speed, the formation of the vortex to isolate high velocity and biological airfoil section, therefore, most of the fluid contact vortex on the surface, only leading to fluid friction model in near wall from sliding friction into rolling friction, due to vortex shock effect, in the biological fluid viscosity resistance is reduced, on the surface of the airfoil section. The TKE dissipation of the turbulent boundary layer is reduced, so the airfoil structure effectively inhibits the total drag.

In addition, not only mantis shrimp has a special bionic nonsmooth surface on its body surface but also the shield scaly structure of shark skin [76] is a special bionic nonsmooth surface. As shown in Figure 15(a), shark, as a cartilaginous fish, is covered by many small toothlike scales or dermal dentate (groove) elements on its body surface. Known as placental scales or dentin [77], dentin consists of an outer ceramic layer and an inner bone-like layer surrounding the pulp cavity. The shield scales can be divided into the basal plate buried in the skin and the spines exposed on the surface of the body. There is a hole in the middle of the lamina with blood vessels and nerves leading into the medullary cavity at the spine. The outermost layer of the shield scale is enamel, and the central medullary cavity is shown in Figure 15(b). The riblet structure on the shield scale can optimize the fluid structure of the fluid boundary layer on the shark body surface, inhibit and delay the occurrence of turbulence, and thus effectively reduce water resistance, reduce energy dependence and consumption, and achieve extremely high swimming speed [76].

Atypical dentin, such as shark tooth shape in different individuals and different parts, shows different characteristics [78]. It is shown in Figure 16 that different shark three-dimensional structures of the single tooth column have different characteristics and can adapt to the different flow fields of the Marine environment; also, the shark scales with tiny ribs are a common characteristic. These ribs are parallel to the direction of swimming, and these shapes enable water to move effectively on the skin surface [29], which is the role of shark rib surface [65, 79]. For a smooth surface, the absolute stress is almost uniform, about 408~738 Pa, but for a single shark skin scale, the value of flow direction is about -580~4700 Pa; the maximum value at the tip is larger than the minimum value at the smooth surface, and the bottom, along the direction, and even the opposite flow direction are much smaller than the smooth surface. The absolute pressure on the skin surface of the shark is also less than that on the smooth surface, so the body surface of the shark presents the effect of reducing drag. In addition, the amount of drag reduction for shark surface grooves depends on the geometry of the ribs, which refers to the height and distance between the ribs. Applying this groove surface to the vehicle can help reduce the drag of the vehicle by up to 8%, which represents a fuel saving of approximately 1.5% [80]. In addition, this form enables the shark to self-clean because the height of the texture increases the water contact angle to nearly 180°.

In addition, some species of fish in the sea with superhydrophobic drag reduction scales differ from the shark's groove, and the fish have hydrophilic chemicals (calcium phosphate, protein, and mucus) and unique layered micro- and nanostructure on the scales, and scales with superhydrophobic surface oils, it also protects the fish from [81] the main causes of oil pollution. Therefore, after an oil spill, fishes in the spill area are rarely affected by oil; in other words, they are not covered by oil, and thus, their swimming is affected [82, 83]. The surface characteristics of fish scales are studied, and it is found that due to the composition and microstructure of fish scales [84, 85], they are superhydrophilic in air, resulting in low adhesion of fish scales to underwater bubbles. The special structure of carp body surface was observed and studied. Its skin was completely covered by a fan scale composed of calcium phosphate skeleton and hydrophilic calcium phosphate protein and a thin layer of mucus. The surface of the scale has many micro papilla several hundred microns in size, as shown in Figures 17(a) and 17(b). The size of the micro papilla gradually decreases from the central region to the margin of the scale. The top and lateral walls of each micro papilla are further decorated with abundant nanoscale “small papules,” as shown in Figure 17(c). These structures make fish scales show superhydrophobicity and play an important role in reducing underwater resistance.

### 3.2. Preparation of Bionic Groove

For the preparation of bionic functional materials, the template technology is basically used to take the natural biological surface as the template and then a bionic copy of the micro-nano structure of the biological surface. Shark skin has long been the focus of bionic drag reduction and antifouling technology. The initial studies of drag reduction properties in aircraft design revealed the unique and complex surface technology of shark skin. Sharklet AFTM microstructural material developed by etching and mold turning is shown in Figure 18.

The Sharklet pattern is scaled down to 30~200 *μ*m according to the shark skin, thus smaller than the ubiquitous grime plank plankton, which reduces spore deposition and overall settlement rate by 86% [86]. However, spores that stick to the shark's surface are not as easily removed by currents as they are on equally smooth surfaces. Segmented blade grooves with a thickness of only 38 *μ*m and a height of 90 *μ*m were produced on acrylic acid using a small-scale computer numerical control mill (CNC) [87]. Toothed and serrated grooves with submillimeter spacing can also be machined on aluminum plates [88]. Another way to make a blade groove is to assemble the separately braided parts together. Stacking assemblies with geometrically adjustable shapes are produced by assembling thin blade elements and spacer elements [89]. By separating the blades, thin blades can be manufactured using the rolling process, eliminating the fear of rolling errors destroying the test plate. Groove spacing is controlled by the sum of tolerances for each blade and its spacer elements, allowing for an increase in overall manufacturing tolerances. The main improvement in this assembly is that it is easy to adjust and reduces the risk of destroying the test plate by rolling error.  Figure 19 shows the assembled grooves. For simulated shark skin grooves and 3d grooves, the complex shapes are usually produced by molds. Micromolding and microstamping have been experimentally evaluated using polymethyl methacrylate (PMMA) as a mold material and silica gel as a replica material [90]. Experiments showed that the accuracy (resolution) of the replicas decreased by 2.2% and 5.5% in the spacing of the stripes, and 8.3% and 5.9% in the height of the stripes. In addition, epoxy resin replicas of shark skin were made using wax sustained-release molds on shark skin and flow tank experiments were carried out in a rectangular pipe section [87].

In addition to preparing the bionic nonsmooth surface through Sharklet pattern, Sun et al. [91] chemically prepared the coating containing the bionic multifunctional zinc oxide nanostructured particles of fish scales, whose shape and structure were similar to the ring scale of Asian aurora. These nanocoatings have adjustable light refraction and reflection, controllable surface wettability, and damped mechanical properties. Huang and Ho use the surface micromachining technology of three layers of polysilicon and two layers of P5G [92] to design and produce a microrib with fish scale pattern, as shown in Figure 20. The results show that fish scales can not only protect fish skin but also have good drag reduction performance. In the field of underwater drag reduction, Bixler and Bhushan [93] studied the surface characteristics of fish scales, shark skin, and plant leaves and developed a new bionic surface, which can reduce oil resistance in closed groove flow, thus reducing resistance and providing self-cleaning performance. Inspired by morphological characteristics of fish skin, Liu et al. [94] prepared zinc oxide and polydimethylsiloxane (PDMS) nets modified with n-octadecane. The experimental results show that ZnO and PDMS-modified mesh have good lipophilicity and hydrophobicity. Studies on drag reduction show that water flow can make semisolid n-octadecane self-texturized, which is similar to compliant fish skin. Therefore, compliant biomimetic materials with regular convex semisolid n-octadecane play an important role in drag reduction. Wu et al. [95] observed and analyzed the microstructure of fish scales and processed micron-level biomimetic fish scale surface with laser engraving machine and polishing machine. The arc-shaped convex groove was engraved on the thick acrylic plate, and the maximum drag reduction rate of the sample at low speed was as high as 2.805%. Dou et al. mixed a variety of compounds and sprayed them on the sample surface and prepared the surface of bionic fish scale by spraying technology [96]. The sample surface is distributed with irregular micron-level caves. The drag reduction test shows that the drag reduction rate of the bionic surface is more and more significant with the increase of the flow rate of the bionic surface, and the drag reduction rate is more than 10% at 13.1 m/s. Therefore, the surface of fish scale has better drag reduction characteristics.

In order to verify the quality and drag reduction efficiency of the bionic groove structure, Luo et al. [97] conducted fluid experiments in water tunnels and obtained the results that the drag reduction rate of the bionic groove can exceed 20% and has satisfactory mechanical properties.

## 4. Synergistic Drag Reduction Analysis of Mucus-Groove

In most cases, the realization of biological drag reduction function is realized by the structure of two or more different parts of the organism or the joint action of different factors [98]. This is because of the structure and form evolved by the organism in order to adapt to the environment and meet the needs of survival, so that it has the maximum adaptability to the environment. Most of the epidermal mucus have a good drag reduction effect, and the V-shaped groove in the scale groove can also have strong drag reduction performance [99–103]. Based on the epidermal morphology of the groove combined with mucus, more than 20% drag reduction can be achieved [97], while the drag reduction of the general groove is 5%-7%. In addition, the viscosity resistance of V-groove [104, 105] is 9.9% lower than that of smooth surface pipe, and the V-groove can save 1%~2% fuel when applied to high-speed hull [89, 106].

### 4.1. Mechanism of Slime-Groove Drag Reduction

By studying the drag reduction mechanism of the loach, it can be found that the loach can not only secrete a layer of lubricating mucus film but also can retain its mucus well by virtue of the groove structure of its skin, so that the mucus will not be rapidly lost through the microstructure of its surface. Therefore, the drag-reducing ability of loach is not only the drag-reducing effect of mucus but also the synergistic drag-reducing effect of mucus and groove structure. The synergistic drag reduction mechanism between mucus and grooves not only has a good drag reduction effect but also the grooves are more conducive to the retention of mucus and make it difficult to fall off. For the resistance reduction of the coating, coating shedding is also an important issue. For example, the layer generally applied to the mechanical surface can indeed produce a good drag reduction effect for a short time, but the mechanical strength of such coating is often poor, and the drag reduction effect cannot last for a long time [34, 36]. So, the conventional way of adding coating to reduce the drag of the vehicle is defective. The slime coating of loach can be preserved for a long time through the groove structure on its scales, and the joint action of slime and groove can reduce drag more effectively than a single way, which also provides ideas for the development of coating drag reduction technology. In addition to the drag reduction of loach surface structure, the flexible deformation mode of loach body also contributes to further increase the drag reduction rate. Loach, due to its self-adaptive characteristics, can always keep the drag reduction rate at a high level within a wide speed range [107], and the maximum drag reduction capacity can even reach 33.63% [108].

In addition, the birch loach avoids or slows down the loss of surface mucus through the tiny groove structure, thus reducing the resistance encountered during swimming through mucus.  Figure 21 shows the microscopic morphology of loach body. Loach surface structure has V-shaped grooves on each scale.  Figure 21(b) shows that the transverse regions of adjacent scales are overlapped.  Figure 21(c) shows a single scale in a shield-like shape. The shape under the scanning microscope is shown in Figure 21(d): annular groove and radial nerve at the bottom, while radial and circular groove at the top. These grooves allow the scales to exhibit great flexibility and elasticity. It can be seen from Figure 21(e) that the height of the V-shaped groove is about 6.5 *μ*m, the distance between each cell is about 5.2 *μ*m, and the apex angle is about 43°.

Wu et al. [95] found in the experiment that when the turbulence speed is 0.66 m/s, the drag reduction efficiency of fish scales reaches the highest level, with the maximum drag reduction rate of 2.805%. After comparing various fish, grass carp also has a similar effect. And it can preserve the mucus.  Figure 22(a) shows that its fish scale structure is similar to that of loach scales [109].  Figure 22(b) shows a crescent-shaped ridge structure at the top, with V-shaped grooves between adjacent ridges. The tip area is exposed to the outside world, and the microstructures distributed along a certain direction are used to reduce the tension of free flow.  Figure 22(c) shows the formation of fluid vortices on the bionic nonsmooth surface. So that the adjacent “crescent” microstructure produced fluid formed stable at low speed “the water” area, thereby significantly reducing the wall shear stress between the fluid and biomimetic surface, it effectively prevents the entry of external turbulence and also prevents the internal low-speed fluid spill, which further led to the formation of reverse flow region and reduced the speed near the surface of the bionic. Therefore, it can not only avoid the transition loss of mucus but also allow the mucus to reduce drag with the groove at the same time.  Figure 23 is the cloud diagram of pressure distribution in simulated turbulence. The unit groove generates a stable low-pressure area, and the high-pressure flow will be absorbed by these areas, which leads to the water film thickness of the bionic surface being larger than that of the smooth surface. Prove that the V-groove can reduce drag and maintain mucus attachment. As the average speed of grass carp during swimming is 65.62 cm/s, it is in low-speed movement. Under low-speed movement, the reduction of resistance is greatly related to contact angle (CA).  Figure 24 shows the graph of the contact angle on the surface of fish scale. From the analysis of the contact angle on the surface of fish scale, it can be seen that the left and right CA values of the measuring point are not equal, that is, *α* and *β* are 10° and 13°, respectively. Therefore, the average value of the CA value can be selected as the final measurement value, which is about 11.5°. At this time, it still has good hydrophilicity, which further proves that diffusion wetting phenomenon and high surface energy exist in the tip area of fish scales. It is also clear from Figures 24(b) and 24(c) that the droplet rapidly diffuses after contacting the microstructure, and the fluidity between the adjacent “crescent-shaped” microstructure slows down significantly, resulting in an adhesion effect on the surface. The surface properties of fish scales change and show hydrophilicity, which can retain liquid (water, surface mucus, etc.) well. Therefore, it helps to reduce the frictional resistance on the surface of fish scales. In addition, by comparing the pressure on the bionic nonsmooth surface with that on the smooth surface, it can be concluded that although the bionic nonsmooth surface produces pressure resistance, the viscous force can still be significantly reduced, so that the total resistance decreases, and the drag reduction effect is significantly stronger than that on the smooth surface [109].

In fact, for rough surfaces, the Wenzel model can be used to find out why diffusion wetting exists, and the calculation formula is [110, 111]

(1) $$\begin{array}{c} \cos\theta_{W}=r\cos\theta_{Y}, \end{array}$$

where *θ*_*W*_ is the apparent contact angle of the model and *θ*_*Y*_ is the intrinsic contact angle. *r* is the roughness of solid surface, where *r* = *S*_*a*_/*S*_*g*_ and *S*_*a*_ and *S*_*g*_ are the actual surface area and apparent surface area, respectively.

### 4.2. Preparation of Groove-Mucus Materials

Femtosecond laser processing is often used in the preparation of biomimetic groove-mucus materials. A femtosecond laser is a micro- plus ultrashort point pulse laser; its pulse duration is very short, only 10^−14^~10^−15^. Although the individual pulse energy of a femtosecond laser is only tens of microjoules to a few millijoules, because all the energy is compressed into a very short pulse duration, the femtosecond laser has extremely high peak power [112].

Yong et al. [113] realized the bionic surface with the interaction of groove and mucus on the silicon surface by a femtosecond laser, as shown in Figure 25(a). A femtosecond laser (50 FS, 1 kHz, 800 nm) with a numerical aperture of 0.45 was focused on for progressive scanning. Periodic micromountain micro-nano composite structures were prepared on the surface of P-type silicon [100], which enhanced the hydrophilicity of silicon surface and realized the superhydrophilicity in air and superhydrophobicity in water. The femtosecond laser-treated underwater superoleophobic silicon exhibits extremely high contact angles and very low viscosity for 1,2-dichloroethane and chloroform. Also using femtosecond laser micromachining technology, transparent underwater ultra-oil-phobic quartz glass was prepared [114], as shown in Figure 25(b). After treatment, a rich nanoparticle structure was obtained on the quartz surface, which was superhydrophilic in air, and the contact angle was close to 0°. Under water, the laser-treated quartz glass not only has excellent superhydrophobic properties but also presents ultrahigh transparency, which can be effectively used in an underwater antifouling optical window. As shown in Figure 25(c), after femtosecond laser treatment, the titanium surface acquired periodic micromountain structure, while the titanium surface was oxidized into titanium dioxide [115]. The rough surface of titanium dioxide not only had superhydrophobicity under water but also its wetting characteristics could be stored by ultraviolet light and darkness. There is a reversible conversion between underwater superhydrophobic and underwater superhydrophilic.

Benefit from different material properties, combined with femtosecond laser microprocessing technology that is super controllable, can be used underwater and is suitable for specific application scenarios such as oil viscosity adjustable underwater superhydrophobic surface oil, anisotropic underwater superhydrophobic surface, adjustable underwater superhydrophobic surface, and transparent underwater superhydrophobic surface. However, the underwater environment limits the application scope of the underwater superhydrophobic surface, so that it cannot work directly in the air application scenario. Although the air superhydrophobic surface also has a certain oil pollution resistance in the air environment, the preparation of the air superhydrophobic surface requires the use of extremely low surface energy materials and the design of a fine chamfering structure, so the preparation of the air superhydrophobic surface by a femtosecond laser is rare [116].

## 5. Expectations

Bionic drag reduction technology plays a very important role in improving energy efficiency and protecting ecology. Bionic drag reduction has gradually become an important hot issue in drag reduction. Slime drag reduction and groove drag reduction technologies have been studied and applied more and more and have attracted more and more attention from scholars. There are still many problems to be solved. On the one hand, the single drag reduction method can play a great role in some specific surface, so that the characteristics of the drag reduction method can be fully exploited to find more drag reduction possibilities, so that the drag reduction technology can play a maximum effect. On the other hand, at present, the theory of the combination of drag reduction technology is constantly improving after year-by-year accumulation. The groove technology can be combined with other drag reduction technologies such as nanopolymer slime and antifouling coating in experiments. The combined drag reduction method has a good research prospect. It is also worth studying how to optimize the traditional groove geometry and design more new groove structures with slime drag reduction technology. At present, the theory of bionic drag reduction is still in the exploratory stage and needs further discussion. The introduction should be succinct, with no subheadings. Limited figures may be included only if they are truly introductory and contain no new results.

## Figures and Tables

**Figure 1:** Histological section of shark [22].

**Figure 2:** (a) Silver light is caused by air trapped between blade surface structures, and (b) surface multicellular, with coronal shape [24].

**Figure 3:** Loach skin map: (a) loach skin sampling map and (b) loach skin cross-section map [30].

**Figure 4:** Mucus secretion [97] and reticular structure [35].

**Figure 5:** Schematic diagram of different reactions of spores and larvae to OEG and PEG surfaces [39].

**Figure 6:** Schematic diagram of (a) soluble matrix, (b) contact leaching, (c) self-polishing copolymer (SPC), and (d) the release coating [48].

**Figure 7:** Self-cleaning schematic diagram of releasing descaling paint [50].

**Figure 8:** Synthesis scheme of gelatin-dopamine conjugate [53].

**Figure 9:** Crosslinking reaction equation between microspheres and acrylic polymer coating [55].

**Figure 10:** Schematic diagram of crosslinked coating microstructure constructed by microspheres [55].

**Figure 11:** Dimer formed by a dimer connected by disulfide bonds in the nonglycosylated region [32].

**Figure 12:** Synthesis diagram of UV-PVA [56].

**Figure 13:** Chemical structure [57].

**Figure 14:** Structure of mantis shrimp [66].

**Figure 15:** Shark shield scale [76]: (a) shield scale domain of shark skin and (b) shield-scale planning structure.

**Figure 16:** Three-dimensional structures of single dentition of different sharks: (a) Galapagos shark, (b) great white shark, (c) whitetip reef shark, and (d) blacktip reef shark [78].

**Figure 17:** Scanning electron microscope (SEM) image of fish scale surface. (c) Inset is oil droplet [85].

**Figure 18:** Drag reduction coating inspired by shark skin antifouling [45].

**Figure 19:** Bionic groove physical picture [89].

**Figure 20:** Extraction of the fissure model: (a) fissure structure: C-scale, D-mucus, and e-epidermis, and (b) chute structure [92].

**Figure 21:** Microscopic morphology of loach body: (a) loach, (b) scale morphology, (c) different positions on the same scale, (d) groove structure, and (e) groove cross section [107].

**Figure 22:** Schematic diagram of water capture defects in (a) geometric structure, (b) crescent-shaped structure, and (c) crescent-shaped microstructure of fish scales [109].

**Figure 23:** Simulated pressure distribution in turbulence [107].

**Figure 24:** Image of fish scale surface contact angle [95].

**Figure 25:** Femtosecond laser preparation of underwater superhydrophobic surfaces of different materials: (a) silicon [113], (b) quartz glass [114], and (c) titanium [115].

**Table 1:** Torque values of the control group and the coating group at different speeds [53].

Speed (m/s)	0.916	1.047	1.178
Control group (mN·m)	1.90	2.50	2.90
Gelatin-DOPA-Fe^3+^ (mN·m)	1.37 ± 0.05	1.83 ± 0.05	2.43 ± 0.02
Gelatin-DOPA-Fe^3+^-GTA-1 (mN·m)	1.07 ± 0.02	1.33 ± 0.02	2.07 ± 0.05
Gelatin-DOPA-Fe^3+^-GTA-2.5 (mN·m)	1.57 ± 0.02	1.93 ± 0.02	2.33 ± 0.02
Gelatin-DOPA-Fe^3+^-GTA-5 (mN·m)	2.03 ± 0.02	2.67 ± 0.05	3.47 ± 0.10
